The article "Overexpression of PIK3R1 Promotes Bone Formation by Regulating Osteoblast Differentiation and Osteoclast Formation" was retracted in 2023. Reasons: signs of a paper mill; suspected computer-generated content; unreliable results or conclusions; lack of ethics approval or compliance.

# Overexpression of PIK3R1 Promotes Bone Formation by Regulating Osteoblast Differentiation and Osteoclast Formation

**DOI:** 10.1155/2021/2909454

**Published:** 2021-10-14

**Authors:** Haitao Zhu, Hua Chen, Degang Ding, Shui Wang, Xiaofeng Dai, Yulong Zhu

**Affiliations:** Department of Orthopedics, Sheyang County People's Hospital, Yancheng City, 224300 Jiangsu, China

## Abstract

In an effort to bolster our understanding of regulation of bone formation in the context of osteoporosis, we screened out differentially expressed genes in osteoporosis patients with high and low bone mineral density by bioinformatics analysis. PIK3R1 is increasingly being nominated as a pivotal mediator in the differentiation of osteoblasts and osteoclasts that is closely related to bone formation. However, the specific mechanisms underlying the way that PIK3R1 affects bone metabolism are not fully elucidated. We intended to examine the potential mechanism by which PIK3R1 regulates osteoblast differentiation. Enrichment analysis was therefore carried out for differentially expressed genes. We noted that the estrogen signaling pathway, TNF signaling pathway, and osteoclast differentiation were markedly associated with ossification, and they displayed enrichment in PIK3R1. Based on western blot, qRT-PCR, and differentiation analysis *in vitro*, we found that upregulation of PIK3R1 enhanced osteoblastic differentiation, as evidenced by increased levels of investigated osteoblast-related genes as well as activities of ALP and ARS, while it notably decreased levels of investigated osteoclast-related genes. On the contrary, downregulation of PIK3R1 decreased levels of osteoblast-related genes and increased levels of osteoclast-related genes. Besides, *in vitro* experiments revealed that PIK3R1 facilitated proliferation and repressed apoptosis of osteoblasts but had an opposite impact on osteoclasts. In summary, PIK3R1 exhibits an osteoprotective effect via regulating osteoblast differentiation, which can be represented as a promising therapeutic target for osteoporosis.

## 1. Introduction

Osteoporosis is featured by low bone mineral density (BMD). Escalating global epidemic of osteoporosis, as a systemic skeletal disorder, because of its association with a serious structural deterioration of bone tissue correlated with risk of (fragility) fractures [1], in older adults [2, 3]. The pattern of pathological consequence in osteoporosis is featured by imbalance between osteoclast differentiation and bone resorption in favor of osteoclast activation [4]. To date, no effective avenues are available for the prevention and treatment of osteoporosis [5].

Osteoclasts are specialized cells that resorb bone and thus are essential for normal skeletal development and remodeling [6]. Unlike lymphocytes and macrophages that are aimed at removing foreign materials, osteoclasts are involved in destructing host tissue. This activity is recognized as a physiologically autoimmune response to bone remodeling. Osteoclast differentiation is a complicated and multistep process [7], being modulated by multiple cytokines (M-CSF, RANKL), growth factors, and hormones [8, 9]. Previous studies have already identified some osteoclast-related transcription factors such as MafB, NFATc1, and MitF [10–12]. Nonetheless, specific molecular mechanism of osteoclast differentiation remains to be fully elucidated. Osteoblasts take a relevant part in bone repairing, which might be a key for an efficient bone formation [13]. The communication between osteoblasts and osteoclasts is observed in each stage of bone remodeling. The molecular mechanism that regulates their interplay is therefore essential in bone cell biology as well as a key process in bone formation and bone homeostasis [14, 15].

The article "Overexpression of PIK3R1 Promotes Bone Formation by Regulating Osteoblast Differentiation and Osteoclast Formation" was retracted in 2023. Reasons: signs of a paper mill; suspected computer-generated content; unreliable results or conclusions; lack of ethics approval or compliance.

PI3K, a heterodimer, consists of a regulatory subunit (p85) and a catalytic subunit (p110), and both of them are expressed in multiple isoforms [16]. In the form of p85*α*, PIK3R1 accounts for 65-75% of intracellular regulatory subunits [17]. PIK3R1 has been recognized as a pivotal mediator in the differentiation of both osteoblasts and osteoclasts that is closely related to bone formation [18]. Currently, a genome-wide association study revealed that PIK3R1 is only enriched in bone formation, but the novel gene has yet to be developed. Moreover, the exact mechanism by which PIK3R1 regulates bone formation remains to be elaborated. Hence, we unraveled that PIK3R1 had an impact on levels of examined osteoblast-related genes and osteoclast-related genes during osteoblasts and osteoclasts differentiation. We manifested that PIK3R1 facilitated differentiation of osteoblast rather than osteoclast. In addition, we identified that PIK3R1 suppressed apoptosis and promoted proliferation of osteoblasts but exerted an opposite effect on osteoclasts. To sum up, PIK3R1 is a regulator of bone formation, which might be a therapeutic target candidate for bone homeostasis.

## 2. Materials and Methods

### 2.1. Data Acquisition and Preprocessing

GSE2208 (Affymetrix Human Genome U133A Array) was downloaded from the Gene Expression Omnibus (GEO, http://www.ncbi.nlm.nih.gov/geo). GSE2208 included 19 women (high BMD: 10; low BMD: 9) (for clinical information, see Supplementary Table 1). After the chip was annotated and the probe ID was mapped to the gene symbol, probes without corresponding gene symbol were excluded. For data preprocessing, *k*-nearest neighbor (KNN) was utilized to fill the missing expression data, followed by logbase2 scaling. Finally, the limma packet (*p* value < 0.05) was normalized. Regarding several probes that only match one gene symbol, the average expression value of probes was computed and regarded as the conclusive gene expression value. For subsequent analysis, differentially expressed genes (DEGs) were obtained.

The article "Overexpression of PIK3R1 Promotes Bone Formation by Regulating Osteoblast Differentiation and Osteoclast Formation" was retracted in 2023. Reasons: signs of a paper mill; suspected computer-generated content; unreliable results or conclusions; lack of ethics approval or compliance.

### 2.2. Enrichment Analysis

By using the clusterProfiler package, functions of DEGs were predicted by Gene Ontology (GO) annotation and Kyoto Encyclopedia of Genes and Genomes (KEGG) enrichment analyses. Thresholds for significant enrichment were *p* value < 0.05 and FDR < 0.05. The results were plotted by “ggplot2,” and only TOP10 significantly enriched terms were depicted.

### 2.3. Cell Culture

Murine monocyte macrophages, RAW264.7, were obtained from the American Type Culture Collection (ATCC, USA). The culture condition was DMEM (Life Technologies, USA) with 10% fetal bovine serum (FBS, Life Technologies, USA), 100 U/ml penicillin, and 100 mg/ml streptomycin (Life Technologies, USA). For osteoclastogenesis, RAW 264.7 cells were treated with M-CSF (50 ng/ml) and RANKL (50 ng/ml) for 7 d. The medium was renewed 3 times (less than 48 h). Cells were cultured in a standard environment.

Murine preosteoblast MC3T3-E1 cells were accessed from the Cell Bank of the Chinese Academy of Sciences (Shanghai, China) and maintained in *α*-MEM (Gibco, USA). All media were added with 10% FBS and 1% penicillin/streptomycin (Invitrogen, USA). Cells were incubated under routine conditions. To induce osteoblast differentiation, MC3T3-E1 cells were cluttered in an osteogenic induction medium containing the standard growth medium, supplemented with 50 mg/l ascorbic acid, 10 mmol/l *β*-glycerophosphate, and 10 nmol/l dexamethasone (Sigma-Aldrich, USA).

### 2.4. Alkaline Phosphatase (ALP) and Alizarin Red S (ARS) Staining

For ALP staining, after formalin fixation (10%) and rinsing twice with PBS (pH 7.4), osteoblasts were maintained with ALP substrate solution, naphthol AS-MX (0.1 mg/ml, Sigma-Aldrich, USA), and fast violet B salt (0.6 mg/ml, Sigma-Aldrich, USA) in 0.1 M Tris-HCl (pH 8.5). In addition, ALP activity was assayed by a LabAssay ALP kit (Wako, Japan) after osteoblasts being rinsed twice with PBS and lysed in Mammalian Protein Extraction Reagent (Pierce, USA) per the specification. Besides, protein quantification using the BCA protein assay kit (Pierce, USA) was implemented under the manufacturer's protocol.

For ARS staining, cells were rinsed twice with PBS and then fixed for 10 min in 2% formaldehyde, followed by 30 min of cell staining with 0.2% ARS solution at 37°C. Each well was rinsed 3 times with distilled water and pictured. The ARS red staining indicated calcium deposition.

The article "Overexpression of PIK3R1 Promotes Bone Formation by Regulating Osteoblast Differentiation and Osteoclast Formation" was retracted in 2023. Reasons: signs of a paper mill; suspected computer-generated content; unreliable results or conclusions; lack of ethics approval or compliance.

### 2.5. RNA Isolation and qRT-PCR

The RNeasy Mini Kit (Qiagen, Germany) was utilized for RNA isolation. Complementary DNA (cDNA) was generated by reversely transcribing RNA on the SuperScript III First-Strand Synthesis System (Life Technologies, Japan). qRT-PCR was conducted on the Step One Plus Real-Time PCR System (Life Technologies, USA) and Fast SYBR Green Master Mix (Life Technologies, USA), with *β*-actin as an internal reference. Primer sequences are listed in Table 1.

### 2.6. Western Blotting

Proteins were extracted from osteoblasts and osteoclasts of mice. Homogenates were extracted in radioimmunoprecipitation assay buffer (Pearce, USA); then, ultrasonic apparatus was used to complete cell lysis. Lysates were subject to 12000 rpm centrifugation at 4°C for 5 min. Subsequently. 50 *μ*g total proteins in each sample were resolved by 10% SDS-PAGE, followed by being electrotransferred onto a PVDF membrane with a semidry blotter (Bio-Rad, USA). Then, the membrane was sealed for 1 h with 5% nonfat dry milk and then incubated overnight with primary antibodies at 4°C, followed by incubating with a secondary antibody. Antibodies used for western blotting are listed in Table 2.

### 2.7. Cell Transfection

Stable knockdown (pLKO.1) PIK3R1 vectors were obtained from Vigene Biosciences (Rockville, USA). Lipofectamine 2000 (Invitrogen, California, USA) was implemented to transfect short hairpin-PIK3R1 (sh-PIK3R1). 24 h later, cells were harvested and subjected to qRT-PCR and western blotting, so as to evaluate transfection efficacy. To generate overexpression-PIK3R1 (oe-PIK3R1) lentivirus, Lipofectamine 2000 was used to transfect 3.6 *μ*g envelope plasmid, 9 *μ*g packaging plasmid, and 12 *μ*g targeting plasmids into cells. 48 h later, lentivirus was obtained and filtered. The sh-NC and oe-NC were controls for sh-PIK3R1 and oe-PIK3R1, respectively.

### 2.8. Assay of Cell Proliferation

After transfection, 1 × 10^4^ cells were seeded into a 96-well plate and 10 *μ*l cell counting kit-8 (CCK-8) reagent (Dojindo Laboratories, Japan) was added at 24, 48, 72, 96, and 120 h. A microplate reader (Thermo Fisher Scientific, USA) was utilized for quantification at 450 nm.

Cells were placed into 48-well plates after transfection. EdU reagent (Sigma-Aldrich, USA) was added to each well at 24 h. 2 h later, cells were subjected to 15 min of fixing with 4% formaldehyde and were treated with 0.5% Triton X-100 for permeabilization. Next, Apollo reaction mixture was dropped into each well and Hoechst 33258 was used for cell staining.

The article "Overexpression of PIK3R1 Promotes Bone Formation by Regulating Osteoblast Differentiation and Osteoclast Formation" was retracted in 2023. Reasons: signs of a paper mill; suspected computer-generated content; unreliable results or conclusions; lack of ethics approval or compliance.

### 2.9. Assay of Cell Apoptosis

First, 2 × 10^4^ cells were rinsed twice in PBS after transfection, followed by resuspension in 100 *μ*l binding buffer. Next, 5 *μ*l Annexin V-FITC and 10 *μ*l PI were used for 15 min of staining with 50 *μ*g/ml RNase A (Sigma-Aldrich, USA), followed by 1 h of cell incubation in an incubator in the dark. A flow cytometer (Becton, Dickinson and Company, USA) was used for cell assay. FlowJo software (Ashland, USA) was utilized for data analysis. The number of viable apoptotic cells was computed by calculating the percentage of Annexin V+/PI- cells. The number of nonviable apoptotic cells was computed by calculating the ratio of Annexin V+/PI+ cells. The number of necrotic cells was computed by calculating the proportion of Annexin V-/PI+ cells. Annexin V-/PI- cells are considered as viable cells [19].

### 2.10. Data Handling

All data were expressed as mean ± SD and processed by GraphPad Prism software v.8.0 (USA). All experiments were repeated 3 times independently, including 3 biological replicates and 3 technical replicates. The Student *t*-test or one-way analysis of variance (ANOVA) with Tukey's post hoc test was performed accordingly. The significant difference was considered when *p* < 0.05.

## 3. Results

### 3.1. Screening of DEGs in Osteoporosis Patients with High and Low BMD

In an effort to probe DEGs in osteoporosis patients with high/low BMD, we analyzed data in the GSE2208 dataset. GSE2208 included 19 women (high BMD: 10; low BMD: 9). Through microarray data processing, 756 DEGs were identified from high and low BMD groups (Figure 1).

### 3.2. Enrichment Analysis on DEGs and Selection of Target Genes

Subsequently, DEGs were subjected to enrichment analysis. The results of GO annotation on 756 DEGs are depicted in Figures 2(a)–2(c). DEGs mainly displayed enrichment in processes relevant to cellular component (CC) such as regulation of RNA splicing, mRNA processing, histone modification, and SMAD protein signal transduction (Figure 2(a)). Regarding biological process (BP), they were mainly enriched in transferring phosphorus-containing groups, nuclear speck, and serine/threonine protein kinase complex (Figure 2(b)). For molecular function (MF), DEGs were mainly enriched in protein C-terminus binding, phosphatase binding, and SMAD binding (Figure 2(c)).

DEGs were then subjected to KEGG signaling enrichment analysis to reveal pathways for these DEGs. As presented in Figure 2(d), DEGs were mainly enriched in apoptosis, estrogen signaling pathway, osteoclast differentiation, and TNF signaling pathway. Next, genes that corresponded to the above pathways were intersected, and FOS, JUN, and PIK3R1 were obtained (Figure 2(e)). Among them, FOS and JUN have already been widely studied in osteoporosis. PIK3R1, which encodes PI3k regulatory subunit alpha, is being nominated as a pivotal mediator in the differentiation of osteoblasts and osteoclasts [18]. Nevertheless, the precise signaling mechanism by which PIK3R1 regulates ossification remains unclear. Thus, PIK3R1 was considered for further studies.

The article "Overexpression of PIK3R1 Promotes Bone Formation by Regulating Osteoblast Differentiation and Osteoclast Formation" was retracted in 2023. Reasons: signs of a paper mill; suspected computer-generated content; unreliable results or conclusions; lack of ethics approval or compliance.

### 3.3. The Impact of PIK3R1 on Osteoblast Differentiation

sh-PIK3R1 was transfected into osteoblasts to decrease PIK3R1 level (Figures 3(a) and 3(b)). ALP and ARS staining were used to assay osteoblastic differentiation level at 7 d and 14 d of transfection, respectively. As illustrated in Figure 3(c), ALP and ARS staining as well as ALP activity assays revealed that knockdown of PIK3R1 notably suppressed osteoblast differentiation. Besides, silencing PIK3R1 restrained mRNA and protein levels of osteoblast-related genes (COL1A1, ALP, RUNX2, SP7, OCN, and OPN) (Figures 3(d) and 3(e)). Through proliferation and apoptosis assays, it was manifested that knockdown of PIK3R1 hindered proliferation and fostered apoptosis of osteoblasts (Figures 3(f)–3(h)).

In addition, a specific lentivirus was used to upregulate PIK3R1 in osteoblasts, so as to validate its role in osteoblast differentiation. qRT-PCR and western blotting were performed to evaluate the efficacy of lentivirus (Figures 4(a) and 4(b)). ALP and ARS staining and ALP activity assays were conducted to assess osteoblastic differentiation capacity. The oe-PIK3R1 group exhibited more significant staining than the oe-NC group, indicating an enhanced ability of osteoblast differentiation by upregulating PIK3R1 (Figure 4(c)). Besides, upregulation of PIK3R1 increased mRNA and protein levels of osteoblast-related genes (COL1A1, ALP, RUNX2, SP7, OCN, and OPN) (Figures 4(d) and 4(e)). Proliferation and apoptosis assays disclosed similar findings that upregulation of PIK3R1 promoted proliferation while suppressed apoptosis of osteoblasts (Figures 4(f)–4(h)).

Collectively, PIK3R1 stimulated the expression of osteoblast-related genes and had a promoting impact on osteoblast proliferation and differentiation.

### 3.4. The Impact of PIK3R1 on Osteoclast Differentiation

As such, PIK3R1 expression was silenced to investigate its role in osteoclast differentiation (Figures 5(a) and 5(b)). The mRNA and protein expression of osteoclast-related genes (TRAF6, c-Fos, NFATc1, TRAP, Cathepsin K) were increased by silencing PIK3R1 (Figures 5(c) and 5(d)). The results disclosed that knockdown of PIK3R1 promoted proliferation and suppressed apoptosis of osteoclasts (Figures 5(e)–5(g)).

The article "Overexpression of PIK3R1 Promotes Bone Formation by Regulating Osteoblast Differentiation and Osteoclast Formation" was retracted in 2023. Reasons: signs of a paper mill; suspected computer-generated content; unreliable results or conclusions; lack of ethics approval or compliance.

In addition, PIK3R1 expression was upregulated to verify its role in osteoclast differentiation. Western blotting and qRT-PCR analyses were performed to examine lentivirus efficacy (Figures 6(a) and 6(b)). As depicted in Figures 6(c) and 6(d), mRNA and protein levels of osteoclast-related genes (TRAF6, c-Fos, NFATc1, TRAP, and Cathepsin K) were hindered by upregulating PIK3R1. Proliferation and apoptosis assays displayed that upregulation of PIK3R1 restrained proliferation while promoted apoptosis of osteoclasts (Figures 6(e)–6(g)). To sum up, PIK3R1 constrained the expression of osteoclast-related genes and showed a repressive impact on osteoclast proliferation and differentiation.

## 4. Discussion

Bone is metabolically active and constantly undergoes remodeling via repetitive cycles of bone formation and bone resorption [20, 21]. Functional impairment of bone remodeling and any imbalance between bone formation and resorption can give rise to ossification reduction or bone homeostasis imbalance, thus resulting in diseases related to bone metabolism such as osteoporosis [22, 23]. Thus, it is pivotal to understand molecular mechanisms underlying modulation of bone remodeling, during osteoblast differentiation and osteoclast formation, which may provide possible targets for the management of osteoporosis and other diseases related to bone metabolism.

Currently, modern high-throughput technology identified a new candidate gene expression profile related to osteoporosis and bone formation [4, 24, 25]. In genetic studies of osteoporosis, Gupta et al. [18] identified several gene candidates, namely, PIK3R1, PRKCH, and SCNN1B, underlying the disease by genome-wide association study, consistent with the method we adopted. First, 756 DEGs were identified by comparing DEGs in 19 women. Next, enrichment analysis was carried out for DEGs to explore relevant functional pathways, which revealed enrichment for multiple pathways, including the estrogen signaling pathway, TNF signaling pathway, and osteoclast differentiation. Besides, numerous studies manifested associations between hsa04915 (estrogen signaling pathway), hsa04668 (TNF signaling pathway), and hsa04380 (osteoclast differentiation) and osteoporosis initiation. For example, estrogen modulates bone metabolism via inducing osteoclast apoptosis and osteoblast level of osteoprotegerin [26]. TNF-*α* suppressed osteoblast differentiation of mesenchymal stem cells and ossification in estrogen-deficiency-induced osteoporosis [27, 28]. ApoE exerted a pivotal role in bone mass maintenance by facilitating osteoblast differentiation via the ERK1/2 pathway [29]. The TNF family has been associated with the pathogenesis of multiple metabolic bone disorders such as osteoporosis [30]. TNF-*α* can induce apoptosis of osteoblasts [31] and synergistically fostered RANKL-induced osteoclast formation, which subsequently contributes to osteoporosis in postmenopausal women [32]. Finally, genes that were involved in the pathways of interest were intersected, and FOS, JUN, and PIK3R1 were obtained. PIK3R1 was identified as a gene related to bone metabolism, but specific mechanism by which PIK3R1 regulates bone metabolism remains underexplored. PIK3R1 was therefore selected for further studies.

The article "Overexpression of PIK3R1 Promotes Bone Formation by Regulating Osteoblast Differentiation and Osteoclast Formation" was retracted in 2023. Reasons: signs of a paper mill; suspected computer-generated content; unreliable results or conclusions; lack of ethics approval or compliance.

PIK3R1 expression in osteoblasts and osteoclasts was explored, and ALP and ARS assays were conducted as proof of osteoblastic differentiation. The results showed that downregulation of PIK3R1 in osteoblasts noticeably decreased ALP and ARS activities while increased osteoclast-related protein levels. These findings demonstrated that PIK3R1 promoted differentiation of osteoblasts and hampered the formation of osteoclasts, consistent with previous studies. For example, Zhu et al. [33] proposed that downregulation of CRYAB expression suppressed BMSC osteoblast differentiation decreases ALP activity, which is consistent with the role of PIK3R1. Moreover, Fan et al. [34] revealed that PIK3R1 is a target of miR-155 and that miR-155 facilitates chondrocyte apoptosis and catabolic activity via targeting the PIK3R1-mediated PI3K/Akt pathway. Mi et al. [35] displayed that miR-7223-5p suppressed proliferation and fostered apoptosis of osteoblasts via targeting PIK3R1. Shuai et al. [36] displayed that PIK3R1 may be a key target of Eucommiae Cortex for osteoporosis by network pharmacology. As such, our findings revealed that downregulation of PIK3R1 is associated with decreased proliferation and augmented apoptosis of osteoblasts, while its upregulation has an opposite effect. While upregulation of PIK3R1 had an impact on the formation of osteoclasts which is able to suppress their proliferation and promote apoptosis, but its downregulation showed an opposite effect. Taken together, PIK3R1 was able to modulate proliferation and apoptosis of osteoblasts and osteoclasts.

Overall, PIK3R1 acts as a regulator in bone formation through modulating osteoblast differentiation and osteoclast formation to maintain bone homeostasis, which could be represented as an encouraging therapeutic target for osteoporosis. Nonetheless, this study failed to probe into the mechanism by which PIK3R1 promoted bone formation. Further investigations are ongoing.

## Figures and Tables

**Figure 1:** Volcano plot of DEGs. Red (logFC > 0 and *p* < 0.05) indicates upregulated DEGs. Green (logFC < 0 and *p* < 0.05) indicates downregulated DEGs.

The article "Overexpression of PIK3R1 Promotes Bone Formation by Regulating Osteoblast Differentiation and Osteoclast Formation" was retracted in 2023. Reasons: signs of a paper mill; suspected computer-generated content; unreliable results or conclusions; lack of ethics approval or compliance.

**Figure 2:** Enrichment analysis on DEGs and selection of target genes: (a) cellular components; (b) biological processes; (c) molecular functions; (d) KEGG pathway analysis; (e) intersection of genes corresponding to enriched pathways (hsa04915: estrogen signaling pathway; hsa04668: TNF signaling pathway; hsa04380: osteoclast differentiation).

**Figure 3:** The impact of PIK3R1 on osteoblast differentiation: (a, b) the transfection efficacy of sh-PIK3R1 determined by qRT-PCR and western blotting; (c) the impact of PIK3R1 downregulation on osteoblast differentiation assessed by ALP and ARS staining; (d) the mRNA levels of osteoblast-related genes assayed via qRT-PCR; (e) the protein levels of osteoblast-related genes measured by western blotting; (f, g) the impact of PIK3R1 downregulation on osteoblast proliferation tested through CCK-8 and EdU; (h) the impact of PIK3R1 downregulation on osteoblast apoptosis measured by flow cytometry; ^∗^*p* < 0.05.

**Figure 4:** The impact of PIK3R1 on osteoblast differentiation: (a, b) the transfection efficacy of oe-PIK3R1 determined by qRT-PCR and western blotting; (c) the impact of PIK3R1 upregulation on osteoblast differentiation assessed by ALP and ARS staining; (d) the mRNA levels of osteoblast-related genes assayed via qRT-PCR; (e) the protein levels of osteoblast-related genes measured by western blotting; (f, g) the impact of PIK3R1 upregulation on osteoblast proliferation tested through CCK-8 and EdU; (h) the impact of PIK3R1 upregulation on osteoblast apoptosis measured by flow cytometry; ^∗^*p* < 0.05.

**Figure 5:** The impact of PIK3R1 on osteoclast differentiation: (a, b) the transfection efficacy of sh-PIK3R1 determined by qRT-PCR and western blotting; (c) the mRNA levels of osteoclast-related genes assayed via qRT-PCR; (d) the protein levels of osteoclast-related genes measured by western blotting; (e, f) the impact of PIK3R1 downregulation on osteoclast proliferation tested through CCK-8 and EdU; (g) the impact of PIK3R1 downregulation on osteoclast apoptosis measured by flow cytometry; ^∗^*p* < 0.05.

**Figure 6:** The impact of PIK3R1 on osteoclast differentiation: (a, b) the transfection efficacy of sh-PIK3R1 determined by qRT-PCR and western blotting; (c) the mRNA levels of osteoclast-related genes assayed via qRT-PCR; (d) the protein levels of osteoclast-related genes measured by western blotting; (e, f) the impact of PIK3R1 upregulation on osteoclast proliferation tested through CCK-8 and EdU; (g) the impact of PIK3R1 upregulation on osteoclast apoptosis measured by flow cytometry; ^∗^*p* < 0.05.

**Table 1:** Primers used in qRT-PCR.

Target gene	Primer (5′-3′)
*β*-Actin	F:5′-CGTCGACAACGGCTCCGGCATG-3′
	R:5′-GGGCCTCGTCACCCACATAGGAG-3′

ALP	F:5′-AATCGGAACAACCTGACTGACC-3′
	R:5′-TCCTTCCACCAGCAAGAAGAA-3′

COL1A1	F:5′-CCTGCTGGCAAGAGTGGT-3′
	R:5′-GCCCTGTTCGCCTGTCT-3′

SP7	F:5′-CCCCATCTCCCTTGACTG-3′
	R:5′-TTCCCCAAAGAGCACATCT-3′

RUNX2	F:5′-TTCTCCAACCCACGAATGCAC-3′
	R:5′-CAGGTACGTGTGGTAGTGAGT-3′

TRAF6	F:5′-AGCCCACGAAAGCCAGAAGAA-3′
	R:5′-CCCTTATGGATTTGATGATGC-3′

c-FOS	F:5′-AAACCGCATGGAGTGTGTTGTTCC-3′
	R:5′-TCAGACCACCTCGACAATGCATGA-3′

NFATc1	F:5′-CCGTTGCTTCCAGAAAATAACA-3′
	R:5′-TGTGGGATGTGAACTCGGAA-3′

TRAP	F:5′-GGGACAATTTCTACTTCACTGGAG-3′
	R:5′-TCAGAGAACACGTCCTCAAAGG-3′

Cathepsin K	F:5′-CCATATGTGGGCCCAGGATG-3′
	R:5′-TCAGGGCTTTCTCGTTCCC-3′

OCN	F:5′-CACACTCCTCGCCCTATTG-3′
	R:5′-TACCTCGCTGCCCTCCT-3′

OPN	F:5′-CCGTGGGAAGGACAGTT-3′
	R:5′-TTGCTCTCATCATTGGCTT-3′

PIK3R1	F:5′-AGCCGCCAGCTCTGATAATA-3′
	R:5′-TCTCCCCAGTACCATTCAGC-3′

The article "Overexpression of PIK3R1 Promotes Bone Formation by Regulating Osteoblast Differentiation and Osteoclast Formation" was retracted in 2023. Reasons: signs of a paper mill; suspected computer-generated content; unreliable results or conclusions; lack of ethics approval or compliance.

**Table 2:** Antibodies used in western blotting.

Proteins (dilution)	Catalogue number	Source
Sp7 (1 : 1000)	ab209484	Abcam
RUNX2 (1 : 1000)	#12556	Cell Signaling Technology
c-Fos (1 : 1000)	#2250	Cell Signaling Technology
NFATc1 (1 : 1000)	#8032	Cell Signaling Technology
PIK3R1 (1 : 1000)	#4257	Cell Signaling Technology
ALP (1 : 1000)	ab229126	Abcam
OCN (1 : 1000)	ab93876	Abcam
OPN (1 : 1000)	ab8448	Abcam
TRAF6 (1 : 2000)	ab33915	Abcam
TRAP (1 : 10000)	ab133238	Abcam
Cathepsin K (1 : 2000)	ab19027	Abcam
*β*-Actin (1 : 1000)	#4970	Cell Signaling Technology
IgG	#14708	Cell Signaling Technology

## Data Availability

The data are not publicly available due to privacy or ethical restrictions.

## Supplementary Materials

Supplementary Materials Supplementary Table 1: clinical information of 19 women included in GSE2208 chip.

## References

[1] Golob A. L., Laya M. B. (2015). Osteoporosis: screening, prevention, and management. *The Medical Clinics of North America*.

[2] Sozen T., Ozisik L., Calik Basaran N. (2017). An overview and management of osteoporosis. *European Journal of Rheumatology*.

[3] Li G., Thabane L., Papaioannou A., Ioannidis G., Levine M. A. H., Adachi J. D. (2017). An overview of osteoporosis and frailty in the elderly. *BMC Musculoskeletal Disorders*.

[4] Zhou Y., Gao Y., Xu C., Shen H., Tian Q., Deng H. W. (2018). A novel approach for correction of crosstalk effects in pathway analysis and its application in osteoporosis research. *Scientific Reports*.

[5] Qaseem A., Forciea M. A., McLean R. M., Denberg T. D., for the Clinical Guidelines Committee of the American College of Physicians (2017). Treatment of low bone density or osteoporosis to prevent fractures in men and women: a clinical practice guideline update from the American College of Physicians. *Annals of Internal Medicine*.

The article "Overexpression of PIK3R1 Promotes Bone Formation by Regulating Osteoblast Differentiation and Osteoclast Formation" was retracted in 2023. Reasons: signs of a paper mill; suspected computer-generated content; unreliable results or conclusions; lack of ethics approval or compliance.

[6] Kitazawa R., Haraguchi R., Fukushima M., Kitazawa S. (2018). Pathologic conditions of hard tissue: role of osteoclasts in osteolytic lesion. *Histochemistry and Cell Biology*.

[7] Franceschetti T., Kessler C. B., Lee S. K., Delany A. M. (2013). miR-29 promotes murine osteoclastogenesis by regulating osteoclast commitment and migration. *The Journal of Biological Chemistry*.

[8] Ikeda K., Takeshita S. (2016). The role of osteoclast differentiation and function in skeletal homeostasis. *Journal of Biochemistry*.

[9] Ge D. W., Wang W. W., Chen H. T., Yang L., Cao X. J. (2017). Functions of microRNAs in osteoporosis. *European Review for Medical and Pharmacological Sciences*.

[10] Weilbaecher K. N., Motyckova G., Huber W. E. (2001). Linkage of M-CSF signaling to Mitf, TFE3, and the osteoclast defect in _Mitf^mi/mi^_ mice. *Molecular Cell*.

[11] Ishida N., Hayashi K., Hoshijima M. (2002). Large scale gene expression analysis of osteoclastogenesis _in vitro_ and elucidation of NFAT2 as a key regulator. *The Journal of Biological Chemistry*.

[12] Kim K., Kim J. H., Lee J. (2007). MafB negatively regulates RANKL-mediated osteoclast differentiation. *Blood*.

[13] Matsuoka K., Park K. A., Ito M., Ikeda K., Takeshita S. (2014). Osteoclast-derived complement component 3a stimulates osteoblast differentiation. *Journal of Bone and Mineral Research*.

[14] Mundy G. R., Elefteriou F. (2006). Boning up on ephrin signaling. *Cell*.

[15] Matsuo K., Irie N. (2008). Osteoclast-osteoblast communication. *Archives of Biochemistry and Biophysics*.

[16] Ueki K., Algenstaedt P., Mauvais-Jarvis F., Kahn C. R. (2000). Positive and negative regulation of phosphoinositide 3-kinase-dependent signaling pathways by three different gene products of the p85*α* regulatory subunit. *Molecular and Cellular Biology*.

[17] Taniguchi C. M., Emanuelli B., Kahn C. R. (2006). Critical nodes in signalling pathways: insights into insulin action. *Nature Reviews. Molecular Cell Biology*.

[18] Gupta M., Cheung C. L., Hsu Y. H. (2011). Identification of homogeneous genetic architecture of multiple genetically correlated traits by block clustering of genome-wide associations. *Journal of Bone and Mineral Research*.

[19] Lin P., Chen F., Sun J. (2015). Mycotoxin zearalenone induces apoptosis in mouse Leydig cells _via_ an endoplasmic reticulum stress-dependent signalling pathway. *Reproductive Toxicology*.

[20] Eastell R., O'Neill T. W., Hofbauer L. C. (2016). Postmenopausal osteoporosis. *Nature Reviews. Disease Primers*.

[21] Kim B. J., Lee Y. S., Lee S. Y. (2018). Osteoclast-secreted SLIT3 coordinates bone resorption and formation. *The Journal of Clinical Investigation*.

The article "Overexpression of PIK3R1 Promotes Bone Formation by Regulating Osteoblast Differentiation and Osteoclast Formation" was retracted in 2023. Reasons: signs of a paper mill; suspected computer-generated content; unreliable results or conclusions; lack of ethics approval or compliance.

[22] Lee W. C., Guntur A. R., Long F., Rosen C. J. (2017). Energy metabolism of the osteoblast: implications for osteoporosis. *Endocrine Reviews*.

[23] Feng X., McDonald J. M. (2011). Disorders of bone remodeling. *Annual Review of Pathology*.

[24] Bian Z., Jin L., Zhang J. (2016). LncRNA--UCA1 enhances cell proliferation and 5-fluorouracil resistance in colorectal cancer by inhibiting miR-204-5p. *Scientific Reports*.

[25] Gao P., Ji L., Zhao T., Gao P. (2015). Identification of transcriptional factors and key genes in primary osteoporosis by DNA microarray. *Medical Science Monitor*.

[26] Osako M. K., Nakagami H., Koibuchi N. (2010). Estrogen inhibits vascular calcification via vascular RANKL System. *Circulation Research*.

[27] Sang C., Zhang Y., Chen F. (2016). Tumor necrosis factor alpha suppresses osteogenic differentiation of MSCs by inhibiting semaphorin 3B via Wnt/*β*-catenin signaling in estrogen-deficiency induced osteoporosis. *Bone*.

[28] Fan J. Z., Yang L., Meng G. L. (2014). Estrogen improves the proliferation and differentiation of hBMSCs derived from postmenopausal osteoporosis through notch signaling pathway. *Molecular and Cellular Biochemistry*.

[29] Noguchi T., Ebina K., Hirao M. (2018). Apolipoprotein E plays crucial roles in maintaining bone mass by promoting osteoblast differentiation via ERK1/2 pathway and by suppressing osteoclast differentiation via c-Fos, NFATc1, and NF-*κ*B pathway. *Biochemical and Biophysical Research Communications*.

[30] Feng X. (2005). Regulatory roles and molecular signaling of TNF family members in osteoclasts. *Gene*.

[31] Wang N., Xin H., Xu P., Yu Z., Shou D. (2019). Erxian decoction attenuates TNF-*α* induced osteoblast apoptosis by modulating the Akt/Nrf2/HO-1 signaling pathway. *Frontiers in Pharmacology*.

[32] Zha L., He L., Liang Y. (2018). TNF-*α* contributes to postmenopausal osteoporosis by synergistically promoting RANKL-induced osteoclast formation. *Biomedicine & Pharmacotherapy*.

[33] Zhu B., Xue F., Li G., Zhang C. (2020). CRYAB promotes osteogenic differentiation of human bone marrow stem cells via stabilizing *β*‐catenin and promoting the Wnt signalling. *Cell Proliferation*.

[34] Fan Z., Liu Y., Shi Z. (2020). MiR-155 promotes interleukin‐1*β*‐induced chondrocyte apoptosis and catabolic activity by targeting PIK3R1-mediated PI3K/Akt pathway. *Journal of Cellular and Molecular Medicine*.

[35] Mi B., Xiong Y., Chen L. (2019). CircRNA AFF4 promotes osteoblast cells proliferation and inhibits apoptosis via the Mir-7223-5p/PIK3R1 axis. *Aging (Albany NY)*.

[36] Shuai Y., Jiang Z., Yuan Q., Tu S., Zeng F. (2020). Deciphering the underlying mechanism of Eucommiae Cortex against osteoporotic fracture by network pharmacology. *Evidence-based Complementary and Alternative Medicine*.

